# A Permissioned Blockchain-Based Clinical Trial Service Platform to Improve Trial Data Transparency

**DOI:** 10.1155/2021/5554487

**Published:** 2021-07-29

**Authors:** Lei Hang, BumHwi Kim, KyuHyung Kim, DoHyeun Kim

**Affiliations:** ^1^Shanghai Normal University Tianhua College, Shanghai 201815, China; ^2^Daegu-Gyeongbuk Research Center, Electronics and Telecommunications Research Institute, Daegu 42994, Republic of Korea; ^3^Department of Computer Engineering, Jeju National University, Jeju 63243, Republic of Korea

## Abstract

The clinical research faces numerous challenges, from patient enrollment to data privacy concerns and regulatory requirements to spiraling costs. Blockchain technology has the potential to overcome these challenges, thus making clinical trials transparent and enhancing public trust in a fair and open process with all stakeholders because of its distinct features such as data immutability and transparency. This paper proposes a permissioned blockchain platform to ensure clinical data transparency and provides secure clinical trial-related solutions. We explore the core functionalities of blockchain applied to clinical trials and illustrate its general principle concretely. These clinical trial operations are automated using the smart contract, which ensures traceability, prevents a posteriori reconstruction, and securely automates the clinical trial. A web-based user interface is also implemented to visualize the data from the blockchain and ease the interaction with the blockchain network. A proof of concept is implemented on Hyperledger Fabric in the case study of clinical management for multiple clinical trials to demonstrate the designed approach's feasibility. Lastly, the experiment results demonstrate the efficiency and usability of the proposed platform.

## 1. Introduction

Clinical trials generate a significant amount of clinical research data to approve new drugs, instruments, and medical or surgical treatments on human participants [1]. During the trial, investigators collect data from the subject at a fixed period, including vital signs, changes to symptoms, side effects, or complications caused by the study drug. Generally, the clinical trial requires collaboration among diverse stakeholders, including regulatory bodies, pharmaceutical companies, clinical sites, and most importantly subjects who participate in the clinical trial [2–4]. Besides, each stakeholder of a clinical trial offers a different set of tools to support all the bases that form the clinical trial infrastructure. The current workflow of clinical trials consists of different steps performed independently of each other [5], as shown in Figure 1. In this model, data is created from disparate sources (smart devices, clinical trial sites), processed, and analyzed by different organizations in their preferred way and format.

It is estimated that near 80% of clinical studies are nonreproducible [6]. The high error rate probably results from human faults, fraud, or misconduct. Clinical trials' data quality can be directly affected by the usual mistakes in data acquisition and transcription [7]. More strict supervision requirements are necessary due to these issues, increasing the further burden of document inspection for clinical research regulators. In general, checking the data quality is not a trivial job. It needs knowledge of both the business domain and data modeling to maintain the data quality at a reasonable level [8].

Blockchain technology can improve clinical trials' quality with better reproducibility and grant both researcher communities with secure data sharing and patient groups with tools guaranteeing their privacy [9]. Many experts and institutes have certificated blockchain technology as an emerging technology to ensure secure data transformation among different stakeholders via a distributed ledger in recent years. A consensus-driven approach is enforced to agree with multiple trustless stakeholders [10, 11]. Blockchain is secure, decentralized info comprised of various peers, which provides storage to record data from an outsized form of entities [12]. It is a series of linked blocks of transferred data between different connected nodes that form the blockchain network. Among various blockchain characteristics, transparency is regarded as the critical characteristic since it enables instant access to data, replicated on all nodes without third parties' interventions [13, 14]. The smart contract [15] is a decentralized application compared with other software types as it resides on the blockchain. The smart contract plays multiple roles, including automating an application's business logic without the involvement of third parties, verifying the predetermined rules of operation, and enforcing obligations on an action if these rules are met [16].

Satoshi Nakamoto invented blockchain in 2008 to serve as the public ledger of the cryptocurrency Bitcoin [17]. As the technology evolves, various applications have been explored other than finance and banking services, for example, in the healthcare sector [18–21]. For example, blockchain-based models for electronic medical records have been proposed that would empower patients to exercise greater ownership of their medical data and enhance data sharing between platforms [22–25]. The characteristics of blockchain technologies such as data transparency and traceability have sparked a boom of the reformation in conventional healthcare organizations, including health data sharing and patient follow-up through transaction trace [26]. It is also indicated that the blockchain technology might also prove useful in supporting or even supplanting the traditional data infrastructure used in clinical trials [27–29]. Immutable clinical trial data recorded using a blockchain may inspire greater confidence in its integrity, resulting in better science, safer medicines, and enhanced public trust in biomedical research. However, most of the existing works either validate blockchain's feasibility in clinical trials or present the conceptual application of blockchain falling short of the specific implementation framework or approach. This paper is aimed at giving a practical way of building blockchain-based applications to offer an efficient, secure, and decentralized trace and track solution for clinical trials and further revolutionize the healthcare industry's developments.

This paper provides the following contributions to make clinical trials transparent and build trust among different stakeholders by using blockchain technologies:

- The structure and functionality of a blockchain-based architecture for managing the clinical trials among various stakeholders are presented. Besides, it demonstrates how pharmaceutical companies and other clinical trial investigators can collect and access clinical data in a secure, distributed manner
- A smart contract is implemented to automate clinical trial-related operations without third party involvement. Besides, various service scenarios related to clinical trials, including subject enrollment, medical data collection, and audit query, are presented to demonstrate how the smart contract can handle these operations
- A proof of concept is implemented using Hyperledger Fabric [30] to demonstrate the proposed solution's usability and effectiveness. This implementation is specified to perform clinical trial-related processes among multiple organizations for multiple clinical trials. Besides, a web-based application is implemented to enable end users to interact with the blockchain network, thereby increasing the operability in practice

The rest of this paper is structured as follows: Section 2 analyzes current issues of clinical trials.  Section 3 overviews some existing studies related to this topic.  Section 4 presents the proposed platform's design, while Section 5 describes the prototype application implemented on top of the designed platform with various snapshots of experiment results.  Section 6 evaluates system performance using multiple performance metrics.  Section 7 evaluates the security of the proposed platform. Lastly, Section 8 concludes the paper and points out research directions in future work.

## 2. Current Issues in Clinical Trials

A steady and efficient influx of medical innovations is critical to ensure that society's emerging medical needs are adequately met. Ongoing research has shown that drug development costs continue to rise with an average of 9% each year [31]. Unfortunately, drug development speed, costs, and success rates have not improved over the years, and in some instances, operating conditions have gotten worse. This has resulted in a situation where success rates for new candidate medicinal products entering clinical development are at an all-time low, with only 11% ultimately making it to the market.

Clinical research generates enormous amounts of trial data every day, which increases the pressures of regulatory agencies to overcome such significant data barriers. Besides, it is becoming evident that legacy data management systems are not strong enough to process and preserve the data extracted from current research studies. These systems lack relevant measures to build trust in the clinical trial industry among consumers and regulators. As a result, the three most giant pharmaceutical conglomerates, Pfizer, Amgen, and Sanofi, all carry out the plan to find an effective way of utilizing blockchain technology in clinical trials, from storing secure data to ultimately reducing research costs [32].

In the past decade, numerous eClinical solutions have emerged, aimed at smoothening trial operations and data management. However, most of these function-specific solutions are unable to communicate with each other. Indeed, most clinical researchers experience issues with keeping track of the status of documents and processes in their clinical operations [33], according to a recent industry-wide survey. Though fully integrated and all-encompassing eClinical platforms exist, in practice, these platforms are only accessible to large pharmaceutical developers for being prohibitively expensive as roughly 65% of trials are performed by academia, hospitals, and smaller industry stakeholders [34]. For regulators who experience difficulty auditing research data, there are no easy and secure way of viewing the complex network of data exchange, no real-time access to results once generated, and no easy way to track data historically [35]. Therefore, the FDA has listed a lack of traceability as one of the top data issues in clinical trials [36].

Patient data accessibility is another major problem in the current clinical trial industry as it involves many different specialty stakeholders and even crosses organizational and national boundaries. Clinical trial stakeholders operate in relative isolation, each applying their software systems, data formats, workflows, and organizational structures. In general, patient data is dispersed across multiple proprietary systems that have no relationship and cooperation with each other, making it exceedingly tough to recruit individuals for trials [37]. However, even worse, when investigators recruit enough patients to initiate a clinical trial, the medical condition of patients for that specific treatment could remain an issue and result in an incorrect study with false positive and false harmful errors.

## 3. Related Works

The clinical trial industry is held in high regard for its pivotal role in advancing human health. The trustworthiness of trial data is primary to modern medical theory and methods but cannot be assured due to various reasons, as described in the previous section. Some clinical trial management systems (CTMS) are used by biotechnology and pharmaceutical industries to manage clinical trials in clinical research. EasyTrial [38] is an online clinical trial management system for administering all clinical trial tasks (operational and logistical), so healthcare professionals can use their time efficiently. All trial data is easily accessible and presented simply and comprehensively from the database. The key features of EasyTrial include complete study overview, security monitoring, study data backup, design of eCRF and questionnaires, management of multiple sites, automatic subject invitation and notification by SMS/email, etc. EDETEK [39] is an innovative clinical solutions company that provides high-quality technology platforms and related clinical services to pharmaceutical, biotechnology, and medical device companies. The clinical data management system enables transforming the study protocol to CRF design and EDC setup, including medical coding and extensive metric dashboards and structure based on CDISC or the sponsor's standards. It also provides various functions such as patient management, site management, clinical data warehousing, and trial supply management. VOXCE [40] is an open-source clinical trial management system that offers complete control of data collection, operation, and analysis. It is built using a subscription model that allows multiple users to be part of that subscription, allowing users to utilize the same libraries and templates, which utilizes questions, sections, and forms. Phoenix CTMS [41] is a modern web application combining database software capabilities in clinical research in one modular system, including patient recruitment, clinical trial management, clinical data management, and electronic data capture. This unmatched feature set is geared to support all operational and regulatory requirements of the clinical front end in academic research, at CROs (Contract Research Organizations) and hospitals conducting clinical studies of any phase. However, these legacy systems are not built for today's complex trials. Even with the best IT support, clinical operation teams still get bogged down in ways that are easily overcome with new technology. For example, duplicative efforts and siloed processes cause inefficiencies and trial delays. The system's maintenance and upgrade raise costs and burdens since these systems are designed in a central architecture. Integration is another challenge that results in low data quality. Moreover, lack of insight can lead to uninformed decisions, and lack of oversight may result in noncompliance.

Blockchain is considered a foundation for improving the clinical research methodology and a step toward better transparency to enhance trust among research institutions, clinical sites, and patient populations. Adopting blockchain technology into the clinical industry brings obvious benefits from secure data tracking and sharing to users' data availability and privacy. A more in-depth exploration of blockchain values in clinical trials remains to be made by exchanging views, ideas, practical problems, and unmet needs between IT and clinical trial specialties. The authors in [42] describe the scope, requirements, system design, and challenges of blockchain technology specific to clinical trials and precision medicine. It is reported that several companies and institutions such as IBM Watson Health and the FDA are developing an initiative to define how blockchain can be used to work across the healthcare data from a variety of sources, including clinical trials, wearables, and electronic health records [43].

The method for using blockchain to provide proof of prespecified endpoints in clinical trial protocols is first reported by Carlisle [44]. The author confirms the use of blockchain as a low-cost, independently verifiable method that could be widely and readily used to audit and verify scientific studies' reliability. The authors in [45] are the first to introduce smart contracts on the Ethereum network to address the data manipulation issues common to clinical trials. The results show that blockchain smart contracts can act as a trusted administrator and provide an immutable record of trial history, including trial registration, protocol, subject registration, and clinical measurements. A hybrid blockchain model is presented to tackle known issues in clinical trials [46]. A public blockchain approach is used for clinical trial recruitment, while a private blockchain approach is used for persistent monitoring. The smart contract feature of Ethereum is also utilized to automate the workflow of clinical trial operations. BlockTrial [47] is another similar system that runs trial-related smart contracts on the Ethereum network. This system allows patients to grant researchers permission to access their data and submit queries for data stored in the blockchain. Scrybe [48] is a blockchain ledger designed for clinical trials, paired with a novel Lightweight Mining (LWM) algorithm, to provide provenance on data with minimal system resource requirements. To demonstrate the superiority of the proposed LWM algorithm, the authors conduct a comprehensive security analysis. The verification results indicate that the algorithm can provide the legal and ethical framework for auditors to validate clinical trials, expedite the research process, and save costs in the process. The authors in [49] present a blockchain system for collecting consent from patients. Each step of the consent collection process appended to the blockchain is attached with a timestamp. In this way, the traceability of the patient's consent is established and maintained unobtrusively.

According to the literature overviewed above, numerous studies have shown that adopting blockchain technology in the clinical trial industry is growing up to a new embranchment and subject field to enhance data privacy, security, and transparency.  Table 1 represents the comparison of the proposed approach with these existing blockchain-based studies. Most of the existing studies either remain just in the design phase without implementation or present a simple implementation. This paper proposes a proof of concept using blockchain to manage trial data and perform trial operations.

## 4. Clinical Trial Service Platform Based on Blockchain

### 4.1. Overview of the Clinical Trial Service Platform

The proposed blockchain-based clinical trial service platform consists of three layers: the physical layer, the service layer, and the application layer. As shown in Figure 2, the bottom layer is the physical layer, comprised of various smart devices for collecting the vital signals from subjects. These devices enable the collection of objective measures of intervention effects in both clinical and remote settings. The service layer adopts the modular design that makes the blockchain network more natural to maintain and extend. This layer encapsulates blockchain technologies' various characteristics into individual modules, including peer-to-peer (P2P) protocol, certificate authority, and consensus. The blockchain network consists of various entities, including distributed ledger, certificate authority, P2P protocol, consensus, and smart contract. The ledger is decentralized storage to maintain the replicated and shared data distributed across the entire network. The smart contract defines the business logic concerning all clinical trial-related operations, such as creating a patient record. The orderer is a particular node performing a consensus algorithm to guarantee the stable operation of the blockchain network and ensure that all peers maintain the data consistency. The event hub is responsible for emitting events whenever a new block is generated or the condition defined in the smart contract is triggered. The functions specified in the smart contract are encapsulated into REST APIs. The external smart devices and applications can integrate with the network by calling these APIs. The application layer describes the way that services provided by the blockchain are visualized to the end user. The blockchain network can be accessed either using responsive web-based applications or native applications on smartphones and tablets.

### 4.2. Roles in the Clinical Trial Service Platform

There are admins, clinical research associates (CRAs), clinical research coordinators (CRCs), principal investigators (PIs), subjects, and smart devices, all of which form the stakeholders of the proposed system, as shown in Figure 3. The pharmaceutical company is the sponsor responsible for creating experiment plans, developing clinical protocols, and preparing instruments and medicines for a clinical trial. The pharmaceutical company is not considered the stakeholder since the CRO provides clinical trial services for the pharmaceutical company on an outsource basis. In this paper, the blockchain management company's admin can set up the network to initiate a clinical trial but cannot perform transactions on the blockchain. Besides, the admin is the network manager of blockchain responsible for user registration and enrollment. CRC and PI are investigators responsible for the conduct of the clinical trial at a trial site. Generally, a clinical trial is conducted by a team of individuals at a clinical site. CRC interacts heavily with subjects, doing things like collecting and entering data. PI is the lead individual of the team responsible for all trial-related activities at the site. Their job is to ensure the protocol is executed precisely as written and may delegate trial-related activities to the clinical team members. CRA is the regulator who works in CRO to review submitted clinical data and those that conduct inspections. The subject is a direct participant of the clinical trial, either as a recipient of the investigational product or as a control. The process of subject enrollment is performed by CRC who has to screen the recruited subjects to see whether they meet the inclusion and exclusion criteria. As the most fundamental part of the clinical trial system, subjects need to transmit the biomedical data collected from smart devices throughout clinical trials. The distributed data lake serves as isolated storage that resides on the blockchain, also known as off-chain data storage. It is used to preserve all clinical data, covering user, device, eCRF, and audit data.

### 4.3. System Architecture of the Clinical Trial Service Platform

As shown in Figure 4, these participants can access the blockchain network through the client applications that can communicate with REST APIs. REST APIs serve as an intermediate between external applications and the blockchain network. The smart contract (SC) is a decentralized application that defines the blockchain network's business logic according to the clinical protocol and automates the clinical trial process. The blockchain network appends an immutable record in the ledger to reflect changes resulting from transactions proposed by external applications, and a transaction response is returned as the response. The key value database (K-V DB) holds the current state of the ledger. Each time a new transaction is agreed upon and added, the K-V DB will update to reflect the latest transaction. The blockchain network comprises multiple channels with various organizations, identities, and data visibility rules. The proposed platform comprises multiple private networks, and each private network is specified for an individual clinical trial. In this way, this platform is appropriate for managing multiple clinical trials, and trial data is shared only between participants within the same network. This paper defines four organizations (blockchain management company, hospital, home, contract research organization), which are business entities that participate in the clinical trial. Each private network consists of four organizations, and each organization holds a copy of the ledger to maintain data consistency.

### 4.4. Smart Contract of the Clinical Trial Service Platform

Figure 5 illustrates the interaction between the application and the blockchain via the smart contract. The smart contract, together with the ledger, forms the blockchain network's heart from a high-level view. External applications invoke the smart contract by requesting the REST API to perform operations on the blockchain network. The smart contract programmatically accesses two distinct parts of the ledger: a transaction log that immutably holds the history of all transactions that ever happened in the blockchain and a world state that records these states' latest value. It can perform actions on the states stored in the world state or query transaction records in the transaction log.

The smart contract is defined in the package, and once deployed to the business network, all transactions are made available to applications. For example, CRC can manage the profile of a subject by invoking the corresponding transaction. Besides, the smart contract provides a specific rule list to evaluate whether or not the user can access or manipulate network resources. For instance, the network administrator is granted permission to perform operations on a network level like starting or stopping the network. Simultaneously, general users are only allowed to access specific resources or perform transactions on them.

The structure of the ledger comprises the transaction log and world state, as shown in Figure 6. This diagram indicates the contents inside the block and the world state associated with the block. A block consists of a header, a data section that contains multiple transactions, and the metadata. The world state stores the current state value of the ledger and changes incessantly against the updated state value, such as when a new subject is created or the subject information is modified. The world state provides rich query support that is flexible and efficient against large index data stores when users want to query the actual data value instead of the keys. The world state can significantly improve the transaction processing throughput since it is unnecessary to traverse the overall transaction log.

### 4.5. Identity Management of the Clinical Trial Service Platform

Public Key Infrastructure (PKI) is aimed at facilitating the secure transfer of information for the clinical trial's network activities. In this paper, the PKI architecture utilizes certificate authorities (CA) responsible for the registration and issuance of digital certificates, as shown in Figure 7. The digital certificate certifies the ownership of a public key by the named subject of the certificate. All participants in the network (e.g., CRC, PI, and CRA) use the issued certificate to certify themselves in the messages they exchange in the network. This approach allows all participants to rely upon the digital signature made about the private key that corresponds to the issued certificate. Recipients of digitally signed messages can verify the received message's origin and integrity by checking whether the signature is valid with the sender's public key. The certificate database provides storage to preserve information about issued certificates, such as the status and validity period. The Certificate Revocation List (CRL) is a secure location where invalid certificates are stored and referred. This paper utilizes the X.509 standard [50], which defines the most commonly used public key certificate format.

Figure 8 illustrates the entire process from certificate issuance to validation in CA. The digital certificate is comprised of three elements: plaintext, ciphertext, and encryption method. The plaintext is sent to CA, which signs the certificate with its private key. Specifically, CA performs a SHA256 function on the plaintext to calculate the hash value H1. Then, CA uses its private key to encrypt the hash value H1 using the RSA algorithm to get the ciphertext *F*′. When validating the digital certificate, the ciphertext *F*′ is decrypted with CA's public key to get a hash value H2. Then, CA performs a SHA256 function again on the plaintext *F* to get the hash value H1. If the value of H1 equals H2, it means the certificate is verified, indicating that the client holds a certificate issued by CA.

Figure 9 represents the process of user registration and enrollment in the clinical trial service platform. When the network is set up, an admin is created as the registrar for the CA. The first step is to enroll the admin using the private and public key generated locally when the network is initialized. The public key is then sent to the CA, which returns an encoded certificate for the admin. The admin sends the blockchain's request to create a new user profile, which contains an id. For example, the participant can send a registration request to the CA with this id, and the CA returns a password accordingly. An enrollment request is then sent to the CA, and the id and password are obtained in the registration process. In response, the CA returns the enrollment certificate (ECert) along with the public key. The ECert is used to request the Transaction Certificate (TCert), and the CA returns the TCert along with the private key for signing the transactions. These credentials are then stored in the wallet, and the user can use them to interact with the blockchain.

## 5. Experiment: Applying the Proposed Platform to Create Prototype Application

### 5.1. Overview of the Prototype Application

We utilize the Hyperledger Composer [51] to implement the blockchain application based on Hyperledger Fabric. All of the fabric network entities ran in the Docker environment hosted in a single Linux virtual machine. The smart contract is written in JavaScript by using the Visual Studio Code and further deployed to all the network peers via composer-cli. A REST server is generated by the composer-rest-server from the deployed business network to be consumed by HTTP or REST clients. The REST server provides create, read, update, and delete (CRUD) operations to manipulate the states of assets or participants and allows transactions to be submitted or retrieved with queries. The data transmission between the external client and the REST is secured using the GitHub Passport middleware; thus, every client must be authenticated before they are permitted to call the REST server's APIs. Hyperledger Explorer [32] is used as a visualization tool to observe blocks, transactions, and other relevant information stored in the ledger. The blockchain web application is implemented with HTML, CSS, and JavaScript. The Apache Tomcat web server ships as a host environment capable of serving the web application. This web application can interact with the fabric network to operate on the resources and perform functions via the REST server's endpoint APIs.

As shown in Figure 10, the fabric network is set up and exploited by eight organizations with corporately decided and signed agreements. An organization refers to a managed group of members, such as the blockchain management company, home, hospital, and CRO. A single membership service provider (MSP) defines the list of members of an organization, as described in Figure 11. In this paper, the organizations manage their members under MSPs, representing different organizational groups in independent clinical trials. It is worth noting that the different MSPs can be used to present the same organization group. For example, the company organization consists of two MSPs, ORG1.MSP and ORG5.MSP, which represent the same blockchain management company that performs different clinical trials. Organizations R1 and R5, which refer to the blockchain management companies, have been empowered to initialize the network.

Each organization (e.g., organization R1) in channel C1 is connected with a client application that can submit transactions and other organizations within the same channel. Similarly, client applications connected with organizations in channel C2 can perform transactions within channel C2. It is worth mentioning that one organization can also have multiple client applications such as R2 and R6. Each peer in channel C1 keeps the same copy of the ledger L1 while peer nodes in channel C2 keep the same copy of the ledger L2. The network is under the control of policy rules specified in network configuration (NC), governed by R1 and R5. Channel C1 is governed in terms of the rules defined by channel policy CP1.

Similarly, channel C2 is governed in terms of the rules defined by channel policy CP2. The ordering service supports applications in both channels and orders transactions into blocks. Besides, each of the eight organizations has a preferred CA.

### 5.2. Smart Contract Implementation

The smart contract is modeled and packaged as a compressed business network definition, consisting of participants, assets, and transactions. Figures 12 and 13 describe the unified class diagram of participant and asset definition, respectively. In this business network, a participant or an asset defined in the business network will generate a corresponding instance founded in the model.

Table 2 describes the defined transactions in the smart contract. The participant is the individual (e.g., CRC and CRA) who enrolls in the business network. The asset represents either a tangible property (e.g., pillbox) or intangible data (e.g., eCRF pillbox data and eCRF BGM data). A participant proposes transactions to operate against a specified resource, such as modifying the participant's info. The prototype application supports four types of operations (read, create, update, delete) that the transaction can perform on the particular network resource. ALL is a particular term to determine that the transaction supports all operations. For example, the user can have full and unhindered access to its profile. Once the smart contract is deployed to the blockchain network, all transactions described in the smart contract are made available to applications.

We specify various access control rules to allow or deny access to resources depending on the user's identity, bound to a specific participant. As shown in Algorithm 1, the description states the rule in plain language; participant defines the type of participant affected by the rule, resource defines the type of resource affected by the rule, condition defines the condition that triggers the rule, action describes the permission type (ALLOW or DENY), and the operation is the action allowed or denied by the rule. For example, the CRC has full operation permissions on the subject while the CRA can only read its profile.

Table 3 presents the sample list of some REST API endpoints used to call transactions provided by the smart contract. Each API contains a URI and verbs such as GET, POST, PUT, and DELETE. The URI specifies the endpoint path, and the verb presents the specific operation to be performed on the resource.

### 5.3. Service Scenario of the Clinical Trial Service Platform

The proposed platform contains ten different service scenarios in the clinical trial. The first scenario, referred to as *user registration and enrollment*, shows that the admin can create the user profile for each participant, as shown in Figure 14. This operation requires the admin to log onto the network before PI, CRC, and CRA can register their identity and enroll in the CA certificate system.  Figure 15 illustrates the second scenario, *user profile management*. The admin can delete the user profile while the PI, CRC, and CRA can only read and update their profiles.  Figure 16 shows the third scenario, *subject profile management*, in which the CRC and PI can create, read, update, and delete a subject while the CRA can only read the subject's profile.  Figure 17 illustrates the fourth scenario, named *device pillbox profile management*, in which the CRC and PI can create, read, update, and delete the device pillbox profile while the pillbox can read its profile.  Figure 18 describes the fifth scenario, *eCRF pillbox data management*, where the pillbox generates the eCRF pillbox data, and the CRC and PI can read the eCRF pillbox data. Figures 19 and 20 show the sixth and seventh scenarios, namely, device BGM profile management and eCRF BGM data management, similar to the fourth and fifth scenarios but with the BGM (blood glucose meter).  Figure 21 describes the eighth scenario, *eCRF PI consult data management*, in which the PI and CRC can create, read, and update the eCRF PI consult data while the CRA can read the eCRF PI consult data.  Figure 22 shows the ninth scenario, *eCRF LAB data management*, in which the PI and CRC can create, read, and update the eCRF lab data while the CRA can read the eCRF lab data.  Figure 23 describes the last scenario, *eCRF CRA audit query*, where the CRA can create, read, and update the eCRF audit query while the CRC and PI can read and update the audit data.

### 5.4. Experiment Results

Figure 24 is a screenshot of the experiment results, presenting the following features (a) REST server interface, (b) eCRF pillbox data, and (c) device pillbox data. The web application authenticates the REST server by navigating to the Github OAuth provider's path. The REST server will redirect the request to GitHub to perform the OAuth authentication flow. After generating the token, Github will redirect back to the REST server and display the access token. The web application then forwards the user requests along with the access token to the REST server. The REST server invokes the smart contract's relevant functions to perform business transactions and returns responses routed back to the web application. For the sake of simplicity, the source code of the prototype application was uploaded to GitHub [52]. The implementation results of our prototype application were videotaped and put on the Internet (https://www.youtube.com/watch?v=Nk3P6PGSksY).

As shown in Figure 25, we can monitor various blockchain data on the browser as Hyperledger Explorer is integrated with the network. Hyperledger Explorer provides a dashboard that gives an overview of the network, such as the number of blocks, transactions, and peer nodes. It also provides an entry to access the detailed information; for example, we can get the details of a transaction in terms of transaction ID, type, creator, channel, and timestamp.

## 6. Performance Evaluation

### 6.1. Evaluation Setup

The prototype application's performance was evaluated using an open-source benchmark simulation tool called Hyperledger Caliper [53]. The experiment was performed using 10 clients in a two-channel network, consisting of 8 organizations with 12 endorser peer nodes in total, as depicted in Table 4. The block size is set to 10 transactions per block, and a new block is formed every 250 ms. The ordering service is in solo mode, which consists only of a single ordering node. The experiment's scripts were specified to target two functions of our prototype: eCRF lab data generation and eCRF lab data query transaction since the user most frequently invokes these two transactions. Ten rounds of tests with a fixed number of transactions were performed by varying the send rate from 100 tps to 1000 tps using different transaction data sizes. The experiment results were averaged to reduce the probability of errors resulting from system overload and network congestion.

### 6.2. Throughput and Network Latency Evaluation

The throughput and latency are two standard performance metrics to evaluate the performance of the blockchain network. The throughput can be further divided into two subcategories concerning the operations to deal with. Read throughput is a specific measure to count the number of read operations completed in a defined period, expressed as read per second (rps). Read throughput is not used as a central performance parameter to measure the blockchain. Most of the systems are typically deployed adjacent to the blockchain to achieve significant reading and query efficiency. Transaction throughput is the rate at which valid transactions are committed by the blockchain in a defined period, expressed as transaction per second (tps). Transaction throughput is not the measure at a single node but across all nodes of the whole network.

(1) $$\begin{array}{c} \text{Read Throughput}=\text{Total readoperations}/\text{timein seconds}, \end{array}$$

(2) $$\begin{array}{c} \text{Transaction Throughput}=\text{Total validtransactions}/\text{totaltime in seconds}. \end{array}$$

Latency can also be separated into two subcategories in terms of the type of operations. Read latency measures the total time to submit a read request and receive the reply. Transaction latency measures the time the entire network takes to validate a transaction, covering the broadcasting time and the allocation time spent by the consensus algorithm.

(3) $$\begin{array}{c} \text{Read Latency}=\text{Response received time}-\text{submission time}, \end{array}$$

(4) $$\begin{array}{c} \text{Transaction Latency}=\text{Confirmation time}-\text{submission time}. \end{array}$$

The transaction throughput increases linearly with the increase in send rate until it flattens out at around 600 tps, the saturation point, as plotted in Figure 26.  Figure 27 plots the evaluation results of the observed transaction latency. The latency rises slowly as the send rate increases; however, it increases significantly when the send rate overs the saturation point.

The evaluation of read throughput and read latency is performed using the same experimental method. As shown in Figure 28, the average read throughput increases linearly as the send rate increases. The graph in Figure 29 shows that average read latency has a relatively small increase with the send rate increase. Unlike the eCRF lab data generation transaction, the throughput of eCRF lab data query transaction increases linearly with the increase in send rate. The reason is that eCRF lab data generation transaction requires much more computing power as this function directly modifies the ledger state. In contrast, eCRF lab data query transaction only performs read operations on the ledger. Moreover, it is evident from the results that the transaction data size has a strong impact on the network performance. The transaction throughput decreases and the transaction latency increases with the growth of the transaction data size.

## 7. Security Verification

### 7.1. Data Privacy

In the prototype application, data privacy is achieved using either channel at the network level or the smart contract's access control rules. Each of these channels represents an isolated clinical trial test in which only authorized participants are allowed to access the data from the ledger; hence, data visibility is limited. The peer on the same channel shares a ledger, and the transaction peer needs to obtain the channel's recognition before it can join the channel and transact with others. The access control rules provide declarative access control over the elements of the business network. By defining access control rules, we can determine which users can perform the specific operation on elements over the network. The prototype application differentiates between access control for elements within a business network and access control for network administrative changes. These rules are evaluated in order, and the first rule whose condition matches determines whether access is granted or denied.

### 7.2. Data Transmission

In the prototype application, the client and the REST server's data transmission is secured using the proper authentication strategy. There are many authentication strategies one can choose from, including a mix of social media such as Facebook, Google, GitHub, and enterprise strategies such as SAML, JSON Web Tokens (JWT), or LDAP. To simplify the implementation, the Github authentication provider can authenticate the client to the REST server before it is permitted to access the business network elements. The service owner (Github account) can grant consent to the client application. The Github authorization server requests consent of the service owner and issues access tokens to clients. The issued token allows the client to access the APIs protected by OAuth2.0. These tokens are stored in a cookie in the local storage of the web browser. The access token is retrieved from the web browser's local storage instead of reauthenticating the user whenever they make a subsequent request. Besides, the business network cards used to connect to the business network are preserved by the REST server itself using the local storage. These business network cards are identities issued by using the Fabric-CA server to register enrollment certificates. The REST server is served in an isolated Docker image, and multiple instances of the REST server are allowed to configure a highly available instance of the persistent data store. It is worth noting that only the network administrator is authenticated to stop, restart, or remove the REST server instance without the application users losing access to the deployed business network over REST.

## 8. Conclusion and Future Work

Blockchain technology has many advantages in security, data protection, and the ability to bridge the disparate system manufacturers, CROs, and study sites. This technology has the benefit of centralization without having all of the data located in one place, making it less vulnerable to external or internal attacks. Few studies focus on a specific implementation approach that guarantees integrity and reliability by using blockchain technology in clinical trials, and there is a lack of practical use cases using blockchain in clinical trials. This paper proposes a clinical trial service platform on blockchain to ensure trial data integrity and secure trial-related services. To demonstrate the proposed approach's usability, a proof of concept is implemented on a permissioned-based network, namely, Hyperledger Fabric. A web-based application is also developed to ease the interaction with the blockchain network. The results demonstrate that smart contracts running on the Hyperledger Fabric network can be used to improve the transparency of data management in clinical trials. The proposed system can improve data integrity and accountability and transparency for the data exchange process and lower transaction costs. Besides, it could contribute to the core technologies in the safe management of trial data and the development of information security services. Furthermore, this study can be extended to a control system to maintain and manage reliable data in any other medical institution. It can be used as a critical technology to develop secure service and data management systems in smart healthcare.

Clinical research generates enormous amounts of trial data every day, which increases the pressures of regulatory agencies to overcome such significant data barriers. In particular, clinical trial management systems require high transaction throughput as well as low processing latency. Our future work will refine the prototype by adopting the blockchain implementation in the production environment.

## Figures and Tables

**Figure 1:** Current clinical trial workflow.

**Figure 2:** The layer-based architecture of the proposed clinical trial service platform.

**Figure 3:** Roles in the proposed clinical trial service platform.

**Figure 4:** The system architecture of the clinical trial service platform.

**Figure 5:** Interaction between application and blockchain via the smart contract.

**Figure 6:** Sample ledger structure.

**Figure 7:** Identity management using certificate authorities.

**Figure 8:** Process of certificate issuance and validation.

**Figure 9:** Execution process of user registration and enrollment.

**Figure 10:** Prototype blockchain network topology.

**Figure 11:** Mapping MSPs to organizations in the prototype.

**Figure 12:** Class diagram showing the participant definition.

**Figure 13:** Class diagram showing the asset definition.

**Figure 14:** User registration and enrollment.

**Figure 15:** User profile management.

**Figure 16:** Subject profile management.

**Figure 17:** Device pillbox profile management.

**Figure 18:** eCRF pillbox data management.

**Figure 19:** Device BGM profile management.

**Figure 20:** eCRF BGM data management.

**Figure 21:** eCRF PI consult data management.

**Figure 22:** eCRF lab data management.

**Figure 23:** eCRF CRA audit query.

**Figure 24:** Screenshot of experiment results.

**Figure 25:** Screenshot of Hyperledger Explorer.

**Figure 26:** Impact of the send rate and transaction data size on blockchain transaction throughput.

**Figure 27:** Impact of the send rate and transaction data size on blockchain transaction latency.

**Figure 28:** Impact of the send rate and transaction data size on blockchain read throughput.

**Figure 29:** Impact of the send rate and transaction data size on blockchain read latency.

**Algorithm 1:** Access control rules in the smart contract.

**Table 1:** Comparison with existing studies based on blockchain.

Name	Framework	Use of smart contract	Network type	Evaluation of security	Proof of concept
[44]	Bitcoin	N/A	Permissionless	No	No
[45]	Ethereum	Yes	Permissioned	No	No
[46]	Ethereum	Yes	Both	No	No
[47]	Ethereum	Yes	Permissioned	No	No
[48]	Bitcoin	Yes	Permissionless	No	No
[49]	N/A	No	Permissioned	Yes	No
Proposed approach	Hyperledger Fabric	Yes	Permissioned	Yes	Yes

**Table 2:** Transaction definitions in the smart contract.

Transaction	Participant	Operation	Resource (participant, asset)
User profile management	Admin	ALL	CRC, CRA, PI
Subject management	CRC, PI	ALL	Subject
Device pillbox profile management	CRC, PI	ALL	Pillbox
Device BGM profile management	CRC, PI	ALL	BGM
eCRF pillbox data management	CRC, PI, pillbox	READ, CREATE	eCRF pillbox data
eCRF BGM data management	CRC, PI, BGM	READ, CREATE	eCRF BGM data
eCRF PI consult data management	CRC, PI, CRA	ALL	eCRF PI consult data
eCRF LAB data management	CRC, PI, CRA	ALL	eCRF lab data
eCRF CRA audit	CRC, PI, CRA	ALL	eCRF audit

**Table 3:** Sample REST API endpoints.

URI	Verb	Description
/api/CreateBgmTransaction	POST	Create device BGM profile
/api/UpdateBgmTransaction	POST	Update device BGM profile
/api/DeleteBgmTransaction	POST	Delete device BGM profile
/api/CreatePillboxTransaction	POST	Create device pillbox profile
/api/UpdatePillboxTransaction	POST	Update device pillbox profile
/api/DeletePillboxTransaction	POST	Delete device pillbox profile
/api/CreateSubjectTransaction	POST	Create subject profile
/api/UpdateSubjectTransaction	POST	Update subject profile
/api/DeleteSubjectTransaction	POST	Delete subject profile
/api/CreateECRFpillboxTransaction	POST	Create eCRF pillbox data
/api/CreateECRFbgmTransaction	POST	Create eCRF BGM data
/api/CreateECRFpiConsultTransaction	POST	Create eCRF PI consult data
/api/CreateECRFlabTransaction	POST	Create eCRF lab data
/api/CreateCRAauditTransaction	POST	Create eCRF audit data
/api/ConfirmECRFpiConsultTransaction	POST	Confirm eCRF PI consult data
/api/ConfirmECRFlabTransaction	POST	Confirm eCRF lab data
/api/system/historian	GET	Retrieve all historian transactions
/api/system/identities/{id}/revoke	POST	Revoke the specified identity
/api/systemidentities/issue	POST	Issue an identity to the specified participant

**Table 4:** Experiment configuration parameters for performance evaluation.

Configurable parameters	Values
Number of clients	10
Number of channels	2
Number of organizations	8
Number of peers	12
Number of transactions	5000
Send rate	100–1000 tps
Transaction data size	50 kb, 250 kb, 500 kb
Block timeout	250 ms
Block size	10 transactions per block
Orderer type	Solo

## Data Availability

The data used to support the findings of this study are available from the corresponding author upon request.

## References

[1] Farrokhyar F., Karanicolas P. J., Thoma A. (2010). Randomized controlled trials of surgical interventions. *Annals of Surgery*.

[2] Bhatt A. (2011). Quality of clinical trials: a moving target. *Perspectives in Clinical Research*.

[3] Gardner W., Lidz C. W., Hartwig K. C. (2005). Authors' reports about research integrity problems in clinical trials. *Contemporary Clinical Trials*.

[4] Rang H. (2013). Bad pharma: how drug companies mislead doctors and harm patients. *British Journal of Clinical Pharmacology*.

[5] Weng C., Li Y., Berhe S. (2013). An Integrated Model for Patient Care and Clinical Trials (IMPACT) to support clinical research visit scheduling workflow for future learning health systems. *Journal of Biomedical Informatics*.

[6] Colhoun H. M., McKeigue P. M., Smith G. D. (2003). Problems of reporting genetic associations with complex outcomes. *Lancet*.

[7] Araujo de Carvalho E. C., Batilana A. P., Claudino W. (2012). Workflow in clinical trial sites & its association with near miss events for data quality: ethnographic, workflow & systems simulation. *PLoS One*.

[8] Ellenberg S. S. (2012). Protecting clinical trial participants and protecting data integrity: are we meeting the challenges?. *PLoS Med*.

[9] (2017). Blockchain for open science and knowledge creation, Bartling, Sönke, & et contributors to living document.

[10] Zheng Z., Xie S., Dai H., Chen X., Wang H. An overview of blockchain technology: architecture, consensus, and future trends.

[11] Lemieux V. L. (2016). Trusting records: is blockchain technology the answer?. *Records Management Journal*.

[12] Underwood S. (2016). *Blockchain beyond bitcoin*.

[13] Jeppsson A., Olsson O. (2017). *Blockchains as a Solution for Traceability and Transparency*.

[14] Golosova J., Romanovs A. The advantages and disadvantages of the blockchain technology.

[15] Szabo N. The idea of smart contracts. http://fon.hum.uva.nl/rob/Courses/InformationInSpeech/.

[16] Nakamoto S. (2019). *Bitcoin: A Peer-to-Peer Electronic Cash System*.

[17] Macrinici D., Cartofeanu C., Gao S. (2018). Smart contract applications within blockchain technology: a systematic mapping study. *Telematics and Informatics*.

[18] Hang L., Choi, Kim (2019). A novel EMR integrity management based on a medical blockchain platform in hospital. *Electronics*.

[19] Jamil F., Hang L., Kim K., Kim D. (2019). A novel medical blockchain model for drug supply chain integrity management in a smart hospital. *Electronics*.

[20] Engelhardt M. A. (2017). Hitching healthcare to the chain: an introduction to blockchain technology in the healthcare sector. *Technology Innovation Management Review*.

[21] Jamil F., Ahmad S., Iqbal N., Kim D.-H. (2020). Towards a remote monitoring of patient vital signs based on IoT-based blockchain integrity management platforms in smart hospitals. *Sensors*.

[22] Gordon W. J., Catalini C. (2018). Blockchain technology for healthcare: facilitating the transition to patient-driven interoperability. *Computational and Structural Biotechnology Journal*.

[23] Iqbal N., Jamil F., Ahmad S., Kim D. (2021). A Novel Blockchain-Based Integrity and Reliable Veterinary Clinic Information Management System Using Predictive Analytics for Provisioning of Quality Health Services. *IEEE Access*.

[24] Zhang P., White J., Schmidt D. C., Lenz G., Rosenbloom S. T. (2018). FHIRChain: applying blockchain to securely and scalably share clinical data. *Computational and Structural Biotechnology Journal*.

[25] Dubovitskaya A. (2017). Secure and trustable electronic medical records sharing using blockchain. *AMIA Annual Symposium Proceedings*.

[26] Roehrs A., da Costa C. A., da Rosa Righi R. (2017). OmniPHR: a distributed architecture model to integrate personal health records. *Journal of Biomedical Informatics*.

[27] Benchoufi M., Ravaud P. (2017). Blockchain technology for improving clinical research quality. *Trials*.

[28] Angeletti F., Chatzigiannakis I., Vitaletti A. The role of blockchain and IoT in recruiting participants for digital clinical trials.

[29] Schöner M. M. (2017). *Blockchain technology in the pharmaceutical industry*.

[30] Cachin C. (2016). Architecture of the hyperledger blockchain fabric. *Workshop on Distributed Cryptocurrencies and Consensus Ledgers*.

[31] Getz K. (2018). Insights into outsourcing practices and oversight effectiveness. *Applied Clinical Trials*.

[32] How blockchain will revolutionise clinical trials. https://pharmaphorum.com/views-and-analysis/how-blockchain-will-revolutionise-clinical-trials-clinical-trials/.

[33] Veeva (2018). *Veeva 2018 Unified Clinical Operations Survey*.

[34] Trialtrove (2016). *Clinical trial landscape: 2015 trial completions*.

[35] van Valkenhoef G., Tervonen T., Brock B. ., Hillege H. (2012). Deficiencies in the transfer and availability of clinical trials evidence: a review of existing systems and standards. *BMC Medical Informatics and Decision Making*.

[36] Hume S., Sarnikar S., Becnel L., Bennett D. (2017). Visualizing and validating metadata traceability within the CDISC standards. *AMIA Summits on Translational Science Proceedings*.

[37] Leroux H., McBride S., Gibson S. (2011). On selecting a clinical trial management system for large scale, multi-centre, multi-modal clinical research study. *Studies in health technology and informatics*.

[38] EasyTrial https://www.easytrial.net/.

[39] EDETEK https://www.edetek.com.

[40] VOXCE https://github.com/trialmanager/voxce.

[41] Phoenix CTMS https://www.phoenixctms.org/.

[42] Shae Z., Tsai J. J. P. On the design of a blockchain platform for clinical trial and precision medicine.

[43] IBM (2017). IBM Watson Health announces collaboration to study the use of blockchain technology for secure exchange of health care data IBM, 11 Jan. http://www-3.ibm.com/press/us/en/pressrelease/51394.wss.

[44] Carlisle B. G. (2014). Proof-of-prespecified-endpoints-inmedical-research-with-the-bitcoin-blockchain. *Web blog post. The Grey Literature*.

[45] Nugent T., Upton D., Cimpoesu M. (2016). Improving data transparency in clinical trials using blockchain smart contracts. *F1000Research*.

[46] Zhuang Y., Hsu C. A hybrid blockchain design for patient recruitments and persistent monitoring for clinical trials.

[47] Maslove D. M., Klein J., Brohman K., Martin P. (2018). Using blockchain technology to manage clinical trials data: a proof-of-concept study. *JMIR medical informatics*.

[48] Benchoufi M., Porcher R., Ravaud P. (2017). Blockchain protocols in clinical trials: transparency and traceability of consent. *F1000Research*.

[49] Brooks R. R. Scrybe: a blockchain ledger for clinical trials.

[50] Cooper D., Santesson S., Farrell S., Boeyen S., Housley R., Polk W. (2008). *RFC 5280: Internet X. 509 Public Key Infrastructure Certificate and Certificate Revocation List (CRL) Profile*.

[51] Gaur N. (2018). *Hands-On Blockchain with Hyperledger: Building decentralized applications with Hyperledger Fabric and Composer*.

[52] Blockchain-based-application-for-clinical-trials. https://github.com/hanglei/Blockchain-based-application-for-clinical-trials.

[53] Hyperledger Caliper. https://www.hyperledger.org/projects/caliper.

